# Correlation between Intestinal Microflora in Irritable Bowel Syndrome and Severity

**DOI:** 10.1155/2022/1031844

**Published:** 2022-05-18

**Authors:** Min Ji, Hua Huang, Xianming Lan

**Affiliations:** The Second People's Hospital of Longgang District, Shenzhen, Guangdong 518112, China

## Abstract

**Background:**

Irritable bowel syndrome (IBS) is a common chronic functional gastrointestinal disease accompanied by changes in intestinal microecology. This study investigated the relationship between gut microbiota and disease severity in patients with irritable bowel syndrome (IBS).

**Methods:**

An observational study was performed on 60 IBS patients (study group) and 20 healthy controls admitted to our hospital from January 2013 to December 2014. Fecal samples were taken after admission to measure intestinal flora including Bifidobacterium, Lactobacillus, Enterobacter, and Enterococcus, and patient blood was collected to determine serum D-lactate and diamine oxidase (DAO) levels. The gut microbiota and serum markers of the two groups were analyzed. The correlation of gut microbiota index levels and serum markers with disease severity, as well as the correlation between gut microbiota index levels and serum markers, were analyzed.

**Results:**

The levels of intestinal *Lactobacillus* and *Bifidobacterium* were lower, while the levels of *Enterococcus* and *Enterobacter* and serum D-lactate were higher in the study group than those in the control group. The levels of intestinal *Lactobacillus* and *Bifidobacterium* were lower, while the levels of *Enterococcus* and *Enterobacter*, serum D-lactate, and DAO were higher in patients with moderate IBS than those in patients with mild IBS. The levels of intestinal *Lactobacillus* and *Bifidobacterium* were lower in patients with severe IBS than those with moderate IBS, while the levels of *Enterococcus* and *Enterobacter*, serum D-lactate, and DAO were higher in patients with severe IBS. There was a significant negative correlation between the levels of *Lactobacillus* and *Bifidobacterium* and disease severity and a significant positive correlation between the levels of *Enterococcus* and *Enterobacter*, D-lactate, and DAO and disease severity. There was a significant negative correlation between the levels of *Lactobacillus* and *Bifidobacterium* and serum D-lactate and DAO, while there was a significant positive correlation between the levels of *Enterococcus* and *Enterobacter* and serum D-lactate and DAO (*P* < 0.05).

**Conclusion:**

Intestinal flora, D-lactate, and DAO were abnormal in IBS patients, and intestinal flora was closely correlated with disease severity, D-lactate, and DAO levels.

## 1. Introduction

Irritable bowel syndrome (IBS) is a common chronic functional gastrointestinal disorder. Most patients experience abdominal distension, abdominal pain, or other abdominal discomfort and changes in defecation habits such as stool property or frequency) [1–4]. IBS has a high incidence in young adults, a long course of disease, and difficult recovery, which poses a great threat to the physical and mental health and quality of life of patients [5–8].

In recent years, the incidence of IBS has continued to increase, but the pathogenesis has not been elucidated. IBS is closely associated with an unhealthy diet, poor mental status, and low mood. In addition, gut dysbiosis and intestinal barrier dysfunction may also be involved in the occurrence and development of IBS [9–11]. However, the current clinical relationship between intestinal flora and IBS has not been widely established.

Therefore, we aimed to investigate the correlation between intestinal microflora content and IBS in IBS patients and healthy individuals.

## 2. Materials and Methods

### 2.1. Study Subjects

A total of 60 IBS patients treated in our hospital from January 2013 to December 2014 were enrolled as the study group. Another 20 healthy subjects who visited the hospital during the same period were selected as the control group. In the study group, there were 23 males and 37 females, aged 18-69 years (mean age 45.15 ± 11.28 years). In terms of disease severity, 21 cases were mild (IBS-SSS score: 75-175), 29 were moderate (IBS-SSS score: 176-300), and 26 were severe (IBS-SSS score>300). In the control group, there were 11 males and 9 females, aged 18-70 years (mean age 44.92 ± 11.35 years). No significant differences in the sex, age, and other clinical data of the two groups were observed (*P* > 0.05).

*Inclusion criteria*. (1) Meeting the diagnostic criteria for IBS (for those in the study group) [12]. They had recurrent abdominal pain or other abdominal discomfort. Patients had at least three seizures per month in the 3 months prior to the start of this study and had at least two of the following symptoms: (a) changes in the fecal characteristics during seizures, (b) changes in the defecation frequency, and (c) symptoms were relieved after defecation. (2) Being capable of functioning independently, with good compliance, and cooperating to complete the investigation. (3) The female is not pregnant or breastfeeding.

*Exclusion criteria*. (1) Treatment with antianxiety and antidepressant drugs, intestinal probiotics, calcium, or vitamin D within 1 month before the start of the study; (2) comorbid hyperthyroidism or diabetes; (3) the presence of other organic diseases of the kidney, liver, or heart; (4) the presence of speech communication disorders and mental system lesions; (5) a history of major abdominal surgery; and (6) the presence of benign and malignant tumors.

### 2.2. Intestinal Flora Detection

After admission, 2-5 g fresh stool samples were collected from all the subjects. Add 9 mL of anaerobic bacteria diluent to the sample, mix well, and dilute to 10^−7^ by 10-fold serial dilution method. Appropriate dilutions were inoculated into Enterococcus, Enterobacter, Lactobacillus, and Bifidobacterium media. Lactobacillus and bifidobacteria were coated with L-shaped coating rods and cultured in a glove anaerobic box for 48-72 h. Enterococci and Enterobacteriaceae are grown in conventional incubators for 24-48 hours. Bacterial identification was performed using a three-level bacterial identification method. Select 30-300 medium for colony counts to determine the number of colonies per gram of specimen. Three plates were evaluated to calculate the average number of each colony in the gut flora.

### 2.3. Detection of D-Lactate and DAO

Four milliliters of blood was collected from all subjects in the fasting state; samples were kept at a room temperature for 30 min, followed by centrifugation (3500 r/min, 15 min. The supernatant was decanted and stored at -80°C. The levels of serum D-lactate and DAO were determined by enzyme-linked immunosorbent assay kit (Wuhan Huamei Bioengineering Co., Ltd., Wuhan, China).

### 2.4. Observation Indexes

(1) The levels of intestinal microflora (Enterococcus, Enterobacter, Lactobacillus, and Bifidobacterium) and serum D-lactate and DAO were compared between the study and control groups. (2) The intestinal flora (Enterococcus, Enterobacter, Lactobacillus, and Bifidobacterium), serum D-lactate, and DAO levels of patients with different conditions were statistically analyzed. (3) The correlation between intestinal microflora index level, serum D-lactate, DAO level, and disease severity was statistically analyzed. (4) The correlation between intestinal microflora index level and serum D-lactate and DAO level was statistically analyzed

### 2.5. Statistical Analysis

The statistical analysis was performed by SPSS22.0 (IBM, USA). The data were expressed as $\bar{x}\pm s$ and analyzed by using the student *t-*test. The enumeration data were expressed as *n* (%) and analyzed by using the Chi-square test. Spearman test was used for correlation analysis. *P* < 0.05 indicated a statistically significant difference.

## 3. Results

### 3.1. Comparison of Intestinal Microflora, Serum D-Lactate, and DAO Levels between the Two Groups

The levels of intestinal Lactobacillus and Bifidobacterium in the study group were lower than those in the control group, while the levels of Enterococcus and Enterobacter and serum D-lactate in the study group were higher than those in the control group (*P* < 0.05; Table 1).

### 3.2. Comparison of Intestinal Microflora, Serum D-Lactate, and DAO Levels in IBS Patients with Different Disease Severity

The levels of intestinal Lactobacillus and Bifidobacterium were lower in patients with moderate IBS than those in patients with mild IBS, while the levels of Enterococcus and Enterobacter, serum D-lactate, and DAO were higher in patients with moderate IBS than those in patients with mild IBS (*P* < 0.05). The levels of intestinal Lactobacillus and Bifidobacterium were lower in patients with severe IBS than those in patients with moderate IBS, while the levels of Enterococcus and Enterobacter, serum D-lactate, and DAO were higher in patients with severe IBS than those in patients with moderate IBS (*P* < 0.05; Table 2).

### 3.3. Correlation between Each Index Level and Disease Severity

There was a significant negative correlation between the levels of Lactobacillus and Bifidobacterium and the degree of disease, while there was a significant positive correlation between the levels of Enterococcus and Enterobacter, D-lactate, and DAO and the degree of disease (*P* < 0.05; Table 3).

### 3.4. Correlation between Intestinal Microflora Index Level and Serum D-Lactate and DAO Levels

There was a significant negative correlation between the levels of Lactobacillus and Bifidobacterium and serum D-lactate and DAO, while there was a significant positive correlation between the levels of Enterococcus and Enterobacter and serum D-lactate and DAO (*P* < 0.05; Table 4).

## 4. Discussion

The types of intestinal microflora in the body are complex and diverse. The dominant bacteria in the intestinal microflora, including Bacteroides and Bifidobacterium, are dependent on the intestinal environment to survive and form a unified system with the intestine [13, 14]. In the normal physiological state, the bacteria exist in the gut in a corresponding proportion to maintain the normal function of the intestinal tract. If gastrointestinal disease occurs, this physiological state is disrupted, resulting in a disorder of the proportion of bacteria in the gut, and eventually a series of symptoms [15, 16]. IBS is a common gastrointestinal disease in which abnormal numbers of intestinal microflora may be an important risk factor [17].

Overgrowth of intestinal bacteria and a decrease in beneficial bacteria are the main causes of IBS [18]. The most common beneficial bacteria in the human body are bifidobacterial, which play an essential role in the intestinal tract. Bifidobacterium can produce nutrients required by the intestine and can significantly promote the growth of the intestinal mucosa. It can also inhibit the growth of intestinal bacterial toxins and reduce the production of harmful substances [19]. Additionally, Bifidobacterium can effectively regulate intestinal function, thus enabling better absorption of required nutrients and resistance to invasion by foreign bacteria [20]. Lactobacillus is also an essential beneficial bacterium that can promote the protective effect of the gastrointestinal mucosa, perform the function of cell phagocytosis, and stimulate the production of cytokines to strengthen the body's immunity. In addition, Lactobacillus can inhibit and resist harmful bacteria and foreign pathogens, thus helping to maintain gastrointestinal function [21] effectively.

Enterobacter and Enterococcus are important pathogens that cause intestinal mucosal injury and immune defense dysfunction in patients with IBS. In addition, enterobacteria grow in the intestine and produce many toxins that weaken gastrointestinal absorption and reduce the body's immunity [22]. This study showed that the levels of intestinal Lactobacillus and Bifidobacterium were lower in the study group than in the control group. In comparison, the levels of Enterococcus and Enterobacter in the study group were higher than those in the control group. There were also significant differences in the levels of different intestinal microflora in IBS patients with varying degrees of disease (*P* < 0.05), indicating that the intestinal microflora of IBS patients was abnormal. This indicates that intestinal microecology is closely related to the onset and progression of IBS.

In addition, the serum D-lactate content is low in the normal body. D-lactate is the product of bacterial metabolism and lysis. Generally, the body does not produce D-lactate and cannot or can only slowly metabolize it. If intestinal barrier function is damaged, intestinal permeability increases and D-lactate produced by intestinal bacteria can reach the blood circulation through the intestinal mucosa. Therefore, serum D-lactate content can reflect the degree of intestinal mucosal damage and permeability. DAO is an intracellular enzyme-containing deaminated putrescine and histamine. It is a catabolic enzyme of polyamines such as histamine, mainly distributed in small intestinal mucosa/cilia epithelial cells of mammals. DAO is highly active, and its activity is closely related to villus height and nucleic acid and protein synthesis of intestinal mucosal cells. If intestinal barrier function is impaired, intestinal mucosal cells are shed into the intestinal lumen. DAO enters lymphatic and blood vessels in the intestinal cell space, resulting in increased DAO content. Therefore, serum DAO can also be used to evaluate the damage and repair of the intestinal barrier [23–25].

In this study, the serum D-lactate and DAO levels in the study group were higher than those in the control group. The increasing range of serum D-lactate and DAO levels continued to increase with the severity of the disease (*P* < 0.05), indicating that the intestinal mucosal function was damaged in IBS patients and that the more serious the disease, the more serious the intestinal mucosal damage. In addition, this study also explored and analyzed the correlation between intestinal microflora index levels and serum D-lactate and DAO levels. The results showed that the levels of Lactobacillus and Bifidobacterium were negatively correlated with serum D-lactate and DAO levels. There was a significant positive correlation between Enterococcus and Enterobacter and serum D-lactate and DAO levels (*P* < 0.05), suggesting that there was also a specific correlation between intestinal microflora disorder and intestinal mucosal injury in IBS patients. Moreover, the more serious the intestinal injury, the lower the levels of Lactobacillus and Bifidobacterium and the higher the contents of Enterococcus and Enterobacter. It is suggested that the treatment plan be formulated or adjusted according to the abnormal content of intestinal microflora, D-lactate, and DAO to ensure the effectiveness and safety of the treatment and ensure practical benefit to patients.

## 5. Conclusions

In conclusion, the intestinal microflora and the levels of D-lactate and DAO are abnormal in patients with IBS. The intestinal microflora is closely related to disease, D-lactate, and DAO levels. A treatment plan can be formulated or adjusted according to clinical practice to ensure the effectiveness of the intervention.

## Figures and Tables

**Table 1:** Comparison of intestinal microflora, serum D-lactate, and DAO levels between two groups ($\bar{x}\pm s$).

Group	Number of cases	Lactobacillus (lg CFU/g)	Bifidobacterium (lg CFU/g)	Enterococcus (lg CFU/g)	Enterobacter (lg CFU/g)	D-lactate (*μ*g/L)	DAO (*μ*g/L)
Study	76	6.49 ± 1.01	6.63 ± 1.26	7.97 ± 1.05	9.11 ± 0.76	14.79 ± 4.56	15.59 ± 5.61
Control	76	7.35 ± 1.18	7.99 ± 1.38	6.86 ± 0.89	7.51 ± 0.83	3.35 ± 1.51	5.64 ± 2.08
*t* value		4.827	6.345	7.030	12.394	20.762	14.498
*P* value		<0.001	<0.001	<0.001	<0.001	<0.001	<0.001

**Table 2:** Comparison of intestinal microflora, serum D-lactate, and DAO levels in IBS patients with different conditions ($\bar{x}\pm s$).

Severity	Number of cases	Lactobacillus (lg CFU/g)	Bifidobacterium (lg CFU/g)	Enterococcus (lg CFU/g)	Enterobacter (lg CFU/g)	D-lactate (*μ*g/L)	DAO (*μ*g/L)
Mild	21	7.21 ± 1.10	7.81 ± 1.15	6.96 ± 0.93	7.70 ± 0.79	8.62 ± 3.55	7.71 ± 4.14
Moderate	29	6.41 ± 1.01	6.70 ± 1.26	7.88 ± 1.05	9.08 ± 0.76	15.01 ± 4.56	16.11 ± 5.61
Severe	26	5.87 ± 0.88	6.01 ± 0.92	8.83 ± 1.03	9.89 ± 0.88	18.96 ± 5.35	19.97 ± 6.33
*t/P* value (mild vs. moderate)		2.663/0.011	3.187/0.003	3.205/0.002	6.233/0.000	5.349/0.000	5.805/0.000
*t*/*P* value (moderate vs. severe)		2.103/0.040	2.296/0.026	3.380/0.001	3.663/0.000	2.911/0.005	2.398/0.020

**Table 3:** The correlation between each index level and the disease condition.

Project		Lactobacillus	Bifidobacterium	Enterococcus	Enterobacter	D-lactate	DAO
The severity of IBS	*r* value	-0.559	-0.570	0.541	0.615	0.580	0.579
	*P* value	<0.001	<0.001	<0.001	<0.001	<0.001	<0.001

**Table 4:** Correlation analysis of intestinal microflora index levels with serum D-lactate and DAO levels.

Project		Lactobacillus	Bifidobacterium	Enterococcus	Enterobacter
D-lactate	*r* value	-0.532	-0.568	0.620	0.581
	*P* value	<0.001	<0.001	<0.001	<0.001
DAO	*r* value	-0.591	-0.577	0.594	0.631
	*P* value	<0.001	<0.001	<0.001	<0.001

## Data Availability

The authors confirm that the data supporting the findings of this study are available within the article.
